# Collaborative Filtering Recommendation of Music MOOC Resources Based on Spark Architecture

**DOI:** 10.1155/2022/2117081

**Published:** 2022-03-07

**Authors:** Lifu Wang

**Affiliations:** Music Conservatory, Shandong University of Arts, Jinan 250000, China

## Abstract

With the rapid development of MOOC platforms, MOOC resources have grown substantially, causing the problem of information overload. It is difficult for users to select the courses they need from a large number of MOOC resources. It is necessary to help users select the right music courses and at the same time make the outstanding music courses stand out. Recommendation systems are considered a more efficient way to solve the information overload problem. To improve the accuracy of the recommendation results of music MOOC resources, a mixed collaborative filtering recommendation algorithm based on Spark architecture is proposed. First, the user data and item data are modeled and scored by the collaborative filtering algorithm, then the tree structure of the XGBoost model and the features of regular learning are combined to predict the scores, and then the two algorithms are mixed to solve the optimal objective function to obtain the set of candidate recommendation data. Then, the frog-jumping algorithm is used to train the weighting factors, and the optimal combination of weighting factors is used as the training result of the samples to realize the data analysis of the mixed collaborative filtering recommendation algorithm. The experimental results in the music MOOC resource show that the average absolute error and root mean square error of the proposed method are 0.406 and 1.117, respectively, when the sparsity is 30%, which are lower than those of other existing collaborative filtering recommendation methods, with higher accuracy and execution efficiency.

## 1. Introduction

In recent years, with the rapid development and popularization of the World Wide Web and smart devices, all kinds of information emerge one after another. Faced with surging information, it is difficult for people to efficiently and accurately obtain the information they want from the vast sea of Internet information, which is the problem of information overload [1–5]. Internet giants such as Alibaba, Baidu, and Google all process and generate petabytes of data every day, and the Internet has also moved from the IT (Information Technology) era to the DT (Data Technology) era [6–8].

The recommendation system of Massive Open Online Course (MOOC) based on big data platform has attracted more and more attention from academia and industry. Thanks to the advantages of easy use, low cost (mostly free of charge), wide coverage of people, autonomous learning, and abundant learning resources, MOOC has developed rapidly since its appearance [9–12]. However, with the rapid development of the MOOC platform, the number of courses has greatly increased, and the quality is uneven, which is difficult to guarantee. For users, it is difficult to accurately and efficiently find the part of courses they really like from a large number of courses, but it reduces users' experience and satisfaction with the MOOC platform [13–15]. It is difficult for the course teacher to make the course stand out and reduces the enthusiasm of the course teacher. In the long run, the user growth rate of the MOOC platform will stagnate, and even users will be lost. Quality courses will be increasingly scarce, which will affect the development of the MOOC platform. Therefore, with the development of the MOOC platform, MOOC platform also has the problem of curriculum information overload, especially music MOOC.

In order to solve the problem of information overload, scientists have put forward many solutions. Recommendation system is proved to be an effective tool to solve the problem of information overload. According to the user's past behavior records, it uses algorithms to recommend new items that may be of interest to users to solve the problem of information overload. Commonly used recommendation algorithms mainly include content-based (CB) recommendation algorithm [16], collaborative filtering (CF) algorithm [17], latent factor model (LFM) [18], and hybrid recommendation (HR) algorithm [19]. At present, there are many research studies on personalized recommendation service for dynamic users by collaborative filtering algorithm. For example, Lim et al. [20] applied the CF algorithm to the tourism recommendation system, providing effective tourist routes and scenic spots according to users' preferences and using the user image tag as an assistant for effective recommendation. Wang et al. [21] used the XGBoost algorithm to predict and analyze the churn of Internet customers. These two algorithms are used in both prediction and recommendation systems, but there are few related research studies on combining the two algorithms.

The architecture of the traditional personalized recommendation system cannot effectively store and analyze large datasets, so it cannot guarantee the timeliness and accuracy of the recommendation model. Therefore, it is very important to study a personalized recommendation system that can store and process large datasets. At present, there are many personalized recommendation systems for big data processing, which are basically distributed frameworks. Based on the distributed framework, Soni et al. [22] and others put forward the collaborative filtering algorithm of items based on Hadoop. When recommendation technology is combined with big data technology, the performance of the big data framework will greatly affect the overall recommendation performance. In terms of sparsity and real time, Hadoop, the current mainstream big data platform, is not suitable for low-latency accurate online computing due to its design characteristics. Spark is a new generation of computing framework that emerged in recent two years. The memory-based features make it much better than the MapReduce framework in computing efficiency. From the storage point of view, the HDFS framework in Hadoop ecological environment is mainly used at present. Babu et al. [22] proposed an electronic product recommendation system based on Spark and achieved good running effect. Sundari et al. [23] proposed an integrated sentiment analysis method of mixed collaborative filtering method in a big data environment.

Therefore, this paper attempts to combine the CF algorithm with the Spark platform with faster computing speed to solve the problem of accurate personalized recommendation of music MOOC resources. The research goal is to improve the traditional CF algorithm according to the characteristics of the MOOC platform and use it as the recommendation engine of the Spark system to design a music MOOC recommendation system architecture so that the MOOC platform can provide more accurate music course recommendations to more users in the case of big data. The main work has been completed in two aspects: (1) according to the application scenario characteristics of the music MOOC platform, the distributed Spark recommendation platform architecture is constructed and (2) combining the efficiency of the XGBoost algorithm with the effectiveness of the collaborative filtering algorithm, the dynamic personalized recommendation of users on the big data platform is completed, and the weight factors are optimized by the shuffled frog leading algorithm.

## 2. Distributed Spark Recommendation Platform Architecture

Recommendation systems are generally designed based on specific usage scenarios, such as Amazon Mall push system based on e-commerce, Netflix based on movie and video recommendation, Pandora based on music network radio, and Facebook based on social network. Because the data processed by the bottom layer of the recommendation system is often massive, in order to run stably in the big data environment, the latest big data computing framework Spark is adopted. In Spark architecture, data, machines, and services can be linearly increased, thus providing real-time and reliable recommendations to users [24].

### 2.1. Ideas of Spark Architecture

In order to face massive data, recommendation engines are often designed according to offline and online computing, so as to achieve faster, more reasonable, and more personalized recommendation. The schematic diagram of the calculation method of Spark architecture is shown in Figure 1.

The data of music MOOC resources are huge, and it is characterized by “write once and read many times” in business. In this case, the traditional relational database is not suitable. When designing a Spark-based recommendation system, this paper adopts the scheme of combining HDFS with master-slave node and realizes a high-performance data warehouse to meet the query and analysis requirements of the recommendation system in a big data environment. Specifically, the data required by the recommendation system are stored in HDFS in the form of a master-slave node, and Spark SQL is used to query the data. For master-slave node mode, Spark SQL can use SQL statements to query just like querying database table. In addition, because Spark SQL is based on Spark, it is much faster than Hive. Only the corresponding columns need to be scanned when querying, so this data warehouse design has high performance. The data warehouse design of the master-slave node is shown in Figure 2.

The data in the data warehouse contain three layers: the raw data layer, the offline intermediate layer, and the recommendation result layer. Each layer has its corresponding computation, and the amount of data and computation decreases gradually from the raw data layer to the recommendation result layer.

### 2.2. Overall Platform Architecture

This system adopts Scala language and is implemented based on Spark. Spark is a distributed computing framework for big data, and its running framework consists of Driver and Executor. When we submit tasks to the Spark cluster, the machine will start a JVM virtual machine to run Spark Context, which is called Driver. When the Spark program runs map, reduce, filter, and other operators, the functions in the operators will be submitted to each machine in the cluster for distributed operation, and the process started by each operation node is called the Executor. The distributed big data computing framework is shown in Figure 3.

Two tasks, offline and online computing, are usually run in Spark Executor, in which online computing often caches RDD data of intermediate results in memory to speed up distributed computing. The data calculated by the Executor will be returned to Spark Driver for further online processing. Spark platform architecture is shown in Figure 4.

## 3. Music MOOC Resource Recommendation Based on Mixed Collaborative Filtering

### 3.1. Mixed Collaborative Filtering

In order to improve the effectiveness and accuracy of collaborative filtering results and to strengthen the applicability of the personalized recommendation system, the score of the traditional CF algorithm and the score of the XGBoost recommendation algorithm are weighted. According to their common scoring results, it is regarded as the limited order of personalized recommendation for dynamic users in big data. XGBoost algorithm is a learning system based on tree structure [25]. Compared with commonly used advanced algorithms, such as ant colony algorithm and fish swarm algorithm, the XGBoost algorithm has good scalability and scalability. In the distributed computing of big data, faced with the correspondence of tens of millions of users' data, XGBoost has solved the problems of memory limitation and slow algorithm speed in the time-consuming link of similarity calculation. The following is a scoring model for user data. The specific methods are as follows.

Firstly, a list of users and items is established, and each user *u* corresponds to a database record, which stores the situation of user *u* accessing items in the big data platform. In this record, the number of visits of user *u* to some items *i* can be mined. Understand user preferences according to the number of visits. In the music MOOC platform, when the number of times that two users visit item *i* reaches the set threshold, they are judged as neighboring users. In the big data platform, all items are classified according to similarity. According to the user's access to item *i* in the last time period, the content similar to item *i* is dynamically recommended for the user to access the platform in the next time period.

The predicted rating of item *i* by user *u* in the recommendation system is obtained by averaging the ratings of item *i* by the *k* neighboring users of user *u*. If a neighboring user of user *u* has not had any rating on item *i*, that user is removed as a neighboring user.

(1) $$\begin{array}{c} P_{u,i}=\frac{1}{k}\sum_{v\in N_{u}\cap S\left(i\right)}M_{v,i}, \end{array}$$

where *S*(*i*) denotes all users who have visited item *i* and *M*_*v*,*i*_ denotes the predicted rating of item *i* by the user *v*.

(2) $$\begin{array}{c} P_{u,i}=\frac{\sum_{v\in N_{u}\cap S\left(i\right)}\text{sim}\left(u,v\right)M_{v,i}}{\sum_{v\in N_{u}\cap S\left(i\right)}\left|\text{sim}\left(u,v\right)\right|}, \end{array}$$

where sim(*u*, *v*) represents the similarity between the target user *u* and the user *v* in the adjacent user set *N*_*u*_. Through the similarity calculation method, it is obtained that

(3) $$\begin{array}{c} P_{u,i}={\bar{M}}_{u}\cdot \frac{\sum_{v\in N_{u}\cap S\left(i\right)}\text{sim}\left(u,v\right)\cdot \left(M_{v,i}-{\bar{M}}_{v}\right)}{\sum_{v\in N_{u}\cap S\left(i\right)}\left|\text{sim}\left(u,v\right)\right|},\\ \text{sim}\left(i,j\right)=\frac{i\cdot j}{\left\|i\right\|\left\|j\right\|}, \end{array}$$

where $\bar{M_{u}}$ and $\bar{M_{v}}$ represent the average score of users *u* and *v*, respectively, and the calculation method is shownas follows:

(4) $$\begin{array}{c} {\bar{M}}_{u}=\frac{1}{N\left(I\left(u\right)\right)}\sum_{i\in I_{u}}M_{ui}. \end{array}$$

Take the top *N* music courses with higher prediction scores and recommend them to users. Let CF algorithm be recommended as *T*_1_ and XGBoost model be recommended as *T*_2_, then the calculation method of the scoring result *T* of the mixed recommendation algorithm is as follows:

(5) $$\begin{array}{c} T=aT_{1}+\left(1-a\right)T_{2}. \end{array}$$

In the evaluation of music course *i* by user *u*, let the weight of collaborative filtering algorithm be *α*_*ui*_, the weight of recommendation algorithm of XGBoost model be *β*_*ui*_, and the interference be *e*.

(6) $$\begin{array}{c} P_{ui}=\alpha_{ui}M_{ui}+\beta_{ui}M_{ui}^{'}+e. \end{array}$$

The dataset consisting of *α*_*ui*_ and *β*_*ui*_ is sparse, and most of the data values are 0. In the process of data fitting by algorithm, *α*_*ui*_ and *β*_*ui*_ can be written as *α*_*u*_ and *β*_*u*_. Therefore, formula (6) can be written as

(7) $$\begin{array}{c} P_{ui}=\alpha_{u}M_{ui}+\beta_{u}M_{ui}^{'}+e. \end{array}$$

According to formula (5), we can know that *α*_*u*_+*β*_*u*_=1.

Finally, the highest value of personalized recommendation score of dynamic users is solved, which is transformed into the minimum difference between the actual score value and the predicted score mean. The calculation method is shown as follows:

(8) $$\begin{array}{c} \min_{\alpha_{u},\beta_{u}}=\sum_{R\in S}{\left(M_{u,j}-{\bar{M}}_{u}\right)}^{2}. \end{array}$$

There are four main indexes to measure the recommendation algorithm, namely, precision, recall, mean absolute error (MAE), and root mean square error (RMSE):

(9) $$\begin{array}{c} \text{precision}=\frac{\left|S_{u}\cap S_{u}^{\prime }\right|}{\left|S_{u}\right|},\\ \text{recall}=\frac{\left|S_{u}\cap S_{u}^{\prime }\right|}{\left|S_{u}^{\prime }\right|}, \end{array}$$

where *S*_*u*_ denotes the set of music courses with the highest predicted values using the mixed algorithm and *S*_*u*_′ denotes the set of music courses with the highest ratings for user *u* in the training sample.

(10) $$\begin{array}{c} \text{MAE}=\frac{1}{\left|\text{count}\left(S\right)\right|}\underset{R\in S}{\sum }\left|R_{u,j}-M_{u,j}\right|,\\ \text{RMSE}=\sqrt{\frac{\sum_{R\in S}{\left(R_{u,j}-M_{u,j}\right)}^{2}}{\text{count}\left(S\right)}}, \end{array}$$

where *R*_*u*,*j*_ denotes the actual rating value of music course *j* by user *u*, *M*_*u*,*j*_ denotes the rating value of music course *j* by user *u* after using the recommendation algorithm, and count(*S*) denotes the total number of user rating sets. In this paper, MAE and RMSE are used as the main metrics for recommendation performance evaluation.

### 3.2. Determination of Collaborative Weight Factor

In this paper, shuffled frog leading algorithm [26] is used to optimize the weight factor. Initialize the weight factor as frog swarm, and then perform shuffled frog leading algorithm to solve the weight factor value. In the process of weight factor optimization, the reciprocal of the difference between the predicted value and the actual value is used as the fitness function of the mixed shuffled frog leading algorithm. In the (*t* + 1)-th calculation iteration, the results after the *t*-th iteration are used. The maximum of the frog fitness function is *X*_*b*_(*t*), and the minimum of the frog fitness function is *X*_*w*_(*t*). In order to ensure that the frogs in the group can move closer to the frog with the largest fitness function value, the frog with the smallest fitness function value starts to move continuously, and the moving method is as follows:

(11) $$\begin{array}{c} \Delta_{w}\left(t\right)=\text{rand}\left(\right)\left(X_{b}\left(t\right)-x\left(t\right)\right). \end{array}$$

(12) $$\begin{array}{c} X_{w}\left(t+1\right)=X_{w}\left(t\right)\Delta_{w}\left(t\right),R_{\text{min}}\leq \Delta_{w}\left(t\right)\leq R_{\max}. \end{array}$$

If the value of *X*_*w*_(*t*+1) solved at time *t*+1 is larger than *X*_*w*_(*t*), that is, it has better fitness, then replace *X*_*w*_(*t*) with *X*_*w*_(*t*+1). Otherwise, continue to execute formulas (11) and (12). With regard to frog moving step size, step size factor *C* can be introduced, so the formula for calculating the *i*-th moving distance of the *k*-th frog is as follows:

(13) $$\begin{array}{c} d_{i}=\text{rand}\left(\right)\times \left(X_{b}^{k}-X_{w}^{k}\right)\times C,\\ C=C_{\min}+\frac{i_{\text{now}}}{G_{\text{global}}}\times \left(C_{\text{max}}-C_{\text{min}}\right), \end{array}$$

where *C*_min_ and *C*_max_ are, respectively, the minimum and maximum moving steps of frogs in the current group, which can be set according to the actual situation. *G*_global_ is the sum of the fitness values of all the frogs in the group. *i*_now_ is the number of times the frog moves at the current time.

When the fitness values of all frogs in the group are close to *X*_*b*_(*t*) and the error is within the set threshold, the algorithm iteration stops. Output the frog distribution map at the current moment, which is the optimal solution.

## 4. Experiment and Result Analysis

### 4.1. Experimental Environment and Dataset

This system runs on a Spark cluster with 6 nodes, and the configuration of each node is exactly the same. The operating system of each node is CentOS 6.5 Linux, 32 GB RAM, 2T hard disk, E5645 @ 2.40 GHz 6-Core CPU, Spark version 1.5.1, and 1000 Mbps network card. The main hardware configuration information and software configuration information of the experiment are shown in Tables 1 and 2, respectively.

This paper adopts the dataset of the http://www.cmooc.com website, which mainly includes two datasets: user's course selection record and user's operation log. By analyzing the user's course selection records, we can obtain that the number of users is 120069 and the number of courses is 68, and we can analyze the interaction between users and courses. We can find that, among the total 18 music courses, only a few of the three courses have a large number of students, about 10,000. However, most music courses have a small number of students, and only about 2,000 users attend these courses. It is not difficult to find that the vast majority of users only choose one music course, so the users' course selection is very sparse, and the dataset has obvious cold start problem. In order to facilitate the experiment and avoid the cold start problem, we set the threshold of cold start to 6.

### 4.2. Acceleration Ratio

In order to verify the influence of the Spark platform on the speed of music MOOC resources, the acceleration ratio of Spark recommendation relative to single-machine recommendation is solved.

(14) $$\begin{array}{c} S=\frac{T_{a}}{T_{s}}, \end{array}$$

where *T*_*a*_ and *T*_*s*_ are recommended times for single machine and Spark multinode, respectively.

From the Spark acceleration performance shown in Table 3, it can be seen that when the number of working nodes increases, the Spark acceleration effect becomes more obvious. The larger the sample size, the more significant the influence of the number of working nodes on the speedup ratio. The sample capacity of Data 1 is 12.95 MB, and when the number of working nodes reaches 6, the speedup ratio is only 0.001 higher than that of the single machine. However, when the sample size is 8.03 GB, the speedup ratio increases by 42.907 compared with the single machine, so the Spark platform improves the recommendation efficiency of large-capacity samples and is especially suitable for the recommendation task of large-scale data.

### 4.3. Recommended Speed and Accuracy Analysis

The recommendation time of the recommendation algorithm proposed in this paper is compared between MapReduce architecture and Spark architecture. As shown in Figure 5, it can be seen that Spark architecture takes less time to obtain Top-N recommendation [27] (MOOC recommendation belongs to Top-N recommendation) than MapReduce architecture.

In order to verify the effectiveness of the proposed mixed collaborative filtering recommendation algorithm, it is compared with traditional collaborative filtering recommendation [28], recommendation based on the XGBoost model [21], and recommendation based on Canopy clustering [29]. Each algorithm was randomly repeated 30 times, and the average values of MAE and RMSE were calculated. The comparison results of MAE with different sparsity are shown in Table 4 and Figure 6. The comparative results of RMSE with different sparsity are shown in Table 5 and Figure 7.

From the above experimental results, it can be seen that, with the increasing sparsity, the prediction accuracy of various collaborative filtering recommendations is also increasing. It shows that the realization of these four algorithms is trained under the condition of a large amount of data. If a user's associated data under the MOOC platform is less (sparsity is lower), the effective recommendation of the user's personalized data cannot be completed at this time, which accords with the characteristics of data mining. When there are few user-related feature data, it is difficult to mine valuable data for the user, and it is even more difficult to achieve effective recommendations according to the user's preferences and habits. Under the same sparsity condition, compared with other existing recommendation methods, the MAE performance of the proposed mixed clustering collaborative filtering recommendation is better. The results show that the proposed method significantly improves the accuracy of personalized service recommendation of music MOOC.

## 5. Conclusions

Personalized recommendation service of music MOOC resources enhances users' experience, and users can efficiently obtain effective data of the platform, avoiding searching and searching in massive data. The good experience of personalized service is based on an accurate recommendation algorithm. If the applicability of the recommendation algorithm is not strong, and the service recommended to users is irrelevant to users, it will burden users with junk data and reduce their experience. In this paper, the XGBoost algorithm and CF algorithm are combined to improve the performance of personalized recommendation on the Spark platform. Experiments show that the proposed algorithm has an excellent performance in accuracy and real time and has strong popularization and application value. Further research will be carried out on the problem of excessive differences in subdatasets caused by randomly dividing datasets.

## Figures and Tables

**Figure 1:** The schematic diagram of the calculation method of Spark architecture.

**Figure 2:** Data warehouse design with master-slave nodes.

**Figure 3:** Distributed big data computing framework.

**Figure 4:** Spark platform architecture.

**Figure 5:** Recommended time comparison.

**Figure 6:** MAE comparison results at different sparsity.

**Figure 7:** RMSE comparison results at different sparsity.

**Table 1:** Hardware configuration.

Number	Node name	CPU	Internal storage capacity	Hard disc capacity (TB)
1	Master	E5645 @ 2.40 GHz 6-Core	32 GB RAM	2
2	Slave01	E5645 @ 2.40 GHz 6-Core	32 GB RAM	2
3	Slave02	E5645 @ 2.40 GHz 6-Core	32 GB RAM	2
4	Slave03	E5645 @ 2.40 GHz 6-Core	32 GB RAM	2
5	Slave04	E5645 @ 2.40 GHz 6-Core	32 GB RAM	2
6	Slave05	E5645 @ 2.40 GHz 6-Core	32 GB RAM	2

**Table 2:** Software configuration.

Number	Node name	Operating system	Spark's version
1	Master	CentOS 6.5 Linux	Spark 1.5.1
2	Slave01		
3	Slave02		
4	Slave03		
5	Slave04		
6	Slave05		

**Table 3:** Spark acceleration performance.

Sample sets	Sample set size	Number of nodes involved in the calculation	Acceleration ratio
Data 1	12.95 MB	1	1.000
		3	1.001
		6	1.001

Data 2	656.82 MB	1	1.000
		3	1.013
		6	1.024

Data 3	1.42 GB	1	1.000
		3	6.473
		6	13.139

Data 4	8.03 GB	1	1.000
		3	22.287
		6	43.907

**Table 4:** Comparison results of MAE with different sparsity.

	Sparsity		
	10%	20%	30%
Traditional collaborative filtering	0.594	0.450	0.416
XGBoost	0.582	0.443	0.411
Canopy cluster	0.542	0.421	0.409
Mixed collaborative filtering	0.538	0.418	0.406

**Table 5:** Comparison results of RMSE with different sparsity.

	Sparsity		
	10%	20%	30%
Traditional collaborative filtering	1.420	1.192	1.172
XGBoost	1.330	1.183	1.138
Canopy cluster	1.311	1.166	1.119
Mixed collaborative filtering	1.283	1.160	1.117

## Data Availability

The experimental data used to support the findings of this study are available from the corresponding author upon request.
